The article "Essential Oil of Pinus koraiensis Exerts Antiobesic and Hypolipidemic Activity via Inhibition of Peroxisome Proliferator-Activated Receptors Gamma Signaling" was published in 2013. Journal: Evid Based Complement Alternat Med.

# Essential Oil of *Pinus koraiensis* Exerts Antiobesic and Hypolipidemic Activity via Inhibition of Peroxisome Proliferator-Activated Receptors Gamma Signaling

**DOI:** 10.1155/2013/947037

**Published:** 2013-08-13

**Authors:** Hyun-Suk Ko, Hyo-Jeong Lee, Hyo-Jung Lee, Eun Jung Sohn, Miyong Yun, Min-Ho Lee, Sung-Hoon Kim

**Affiliations:** ^1^College of Oriental Medicine, Kyung Hee University, 1 Hoegi-dong, Dongdaemun-gu, Seoul 130-701, Republic of Korea; ^2^Medical Genomics Research Center, Korea Research Institute of Bioscience and Biotechnology, Daejeon 305-811, Republic of Korea; ^3^College of Life Sciences and Biotechnology, Kyung Hee University, Seoul 130-701, Republic of Korea

## Abstract

Our group previously reported that essential oil of *Pinus koraiensis* (EOPK) exerts antihyperlipidemic effects via upregulation of low-density lipoprotein receptor and inhibition of acyl-coenzyme A. In the present study, we investigated the antiobesity and hypolipidemic mechanism of EOPK using *in vitro* 3T3-L1 cells and *in vivo* HFD-fed rats. EOPK markedly suppressed fat accumulation and intracellular triglyceride associated with downregulation of adipogenic transcription factor expression, including PPAR**γ** and CEBP**α** in the differentiated 3T3-L1 adipocytes. Additionally, EOPK attenuated the expression levels of FABP and GPDH as target genes of PPAR**γ** during adipocyte differentiation. Furthermore, PPAR**γ** inhibitor GW9662 enhanced the decreased expression of FABP and PPAR**γ** and fat accumulation induced by EOPK. To confirm the *in vitro* activity of EOPK, animal study was performed by administering normal diet, HFD, and/or EOPK at the dose of 100 or 200 mg/kg for 6 weeks. Consistently, EOPK significantly suppressed body weight gain, serum triglyceride, total cholesterol, LDL cholesterol, and AI value and increased HDL cholesterol in a dose-dependent manner. Immunohistochemistry revealed that EOPK treatment abrogated the expression of PPAR**γ** in the liver tissue sections of EOPK-treated rats. Taken together, our findings suggest that EOPK has the antiobesic and hypolipidemic potential via inhibition of PPAR**γ**-related signaling.

## 1. Introduction

Obesity as a medical condition of excess body fat caused by an accumulation of adipose tissue mass [1] is tightly associated with various health disorders such as hyperlipidemia, diabetes, and cardiovascular diseases [2]. In obesity, adipocytes accumulate excessive fat and adipocytokine production is disrupted [3, 4]. Adipose tissue development observed in obese individuals is closely related to hypertrophy and hyperplasia, the latter involving proliferation and differentiation of preadipocytes to adipocytes. The peroxisome proliferator-activated receptor (PPAR) and CCAAT/enhancer-binding proteins (C/EBP) families of transcription factors regulate this adipocyte differentiation [5–8]. These transcriptional factors regulate the expression of genes involved in the induction adipocyte phenotypes [5]. 

Pharmaceutical antiobesity drugs are generally developed to loss or control body weight. Although various prescribed or nonprescribed medications have been used for treatment of obesity patients, there is a limitation to apply long-term use because of their severe side effects. Only orlistat (Xenical) has been approved by the FDA for long-term use. Recently, many studies reported antiobesity activity of natural products and suggested the potential as antiobesity agents or their supplements. 

*Pinus koraiensis *(Phylum Pinophyta, Class Pinopsida, Order Pinales, Family Pinaceae) is an evergreen tree found in Korea, China, far eastern Russia, and central Japan. The major bioactive chemicals from *P. koraiensis *include camphene, D-limonene, *α*-pinene, borneol, *β*-pinene, 4-carene, bicyclo-hept-3-ene, 3-carene, *β*-phellandrene, and fencyl [9]. We and others demonstrated the biological efficacies and genotoxicity of essential oil from *P. koraiensis* seed, leaf, nut, and cone [9–13]. However, the biological and biochemical effects of essential oil from *P. koraiensis *have not been reported yet.

Recently, many studies reported that natural products such as *Rhizoma Polygonati falcatum* (RPF) [14],* Boussingaultia gracilis* Miers var. *pseudobaselloides* Bailey [15], Chinese black tea (Pu-erh tea) extract, and gallic acid [16] showed the potential of antiobesity activity *in vitro* or *in vivo*. In the present study, we investigated the antiobesic and hypolipidemic effect of essential oil of *P. koraiensis *SIEB (EOPK) in 3T3-L1 cells by Oil-Red O staining, measuring triglyceride, and analyzing expression levels of adipogenic factors and in high-fat diet-fed rats by measuring body weights and fats, and lipid metabolites.

## 2. Materials and Methods

### 2.1. Preparation of Essential Oil of *P. koraiensis* Leaves (EOPK)

EOPK was prepared using the hydrodistillation method [17]. Driedand pulverized *P. koraiensis* leaves were immersed in distilled water and submitted to steam distillation using an apparatus with a condenser (Hanil Labtech, Seoul, Korea). The distillation continued for 3-4 h at 90°C, and then the volatile compounds contained in the water-soluble fraction were allowed to settle for 20 min. The essential oil layer was separated and purified through microfiltration.

### 2.2. Cell Culture

3T3-L1 preadipocytes were purchased from Korean Cell Line Bank (KCLB). The cells were cultured in Dulbecco's Modified Eagle's Medium (DMEM) with 10% FBS in a humidified atmosphere of 95% air and 5% CO_2_ at 37°C.

### 2.3. Cytotoxicity Assay

The cytotoxicity of EOPK against 3T3-L1 cells was measured by 3-(4,5-dimethyl-2-thiazolyl)-2,5-diphenyl-2H-tetrazolium bromide (MTT) colorimetric assay. The cells were seeded onto 96-well microplates at a density of 1 × 10^4^ cells per well and treated with various concentrations of EOPK (0, 12.5, 25, or 50 *μ*g/mL) for 24 h. MTT working solution was then added to the microplates at 37°C for 2 h, and then MTT extraction buffer (20% SDS and 50% dimethylformamide) was added at 37°C overnight. Optical density (OD) was measured using microplate reader (Sunrise, TECAN, Mannedorf, Switzerland) at 570 nm. Cell viability was calculated by employing the following equation: cell viability (%) = [OD (EOPK) − OD (Blank)]/[OD (Control) − OD (Blank)] × 100.

### 2.4. Differentiation Induction and Oil-Red O Staining

The preadipocyte 3T3-L1 cells were plated onto 6-well plates on day 0 and incubated to confluent status. For adipocyte differentiation, the confluent cells were treated with 1 *μ*M dexamethasone, 1 *μ*g/mL insulin, and 0.5 mM IBMX for 2 days, and the medium was replaced by fresh normal medium only containing 1 *μ*g/mL insulin. On day 8, the differentiated adipocyte cells were cultured in the presence or absence of EOPK (100 *μ*g/mL) for 2 days. The cells were fixed with 2% paraformaldehyde, washed twice with PBS, and finally stained with Oil-Red. After dissolving, cellular-lipid retained Oil-Red O in isopropanol, and adipocyte expression was estimated by measuring OD using microplate reader (Sunrise, TECAN, Mannedorf, Switzerland) at 510 nm.

### 2.5. RT-PCR Analysis

The 3T3-L1 cells were treated with or without EOPK (50 or 100 mg/mL) for 24 h. The total RNA was extracted by using TRIzol reagent (Invitrogen, Carlsbad, CA, USA) according to the manufacturer's instructions. cDNA was synthesized from 1 *μ*g of total RNA and subjected to PCR reaction by using a SuperScript One-Step reverse transcription-PCR (RT-PCR) kit (Invitrogen, Carlsbad, CA, USA). The PCR conditions were 30 cycles of 94°C for 30 s, 57°C for 30 s, and 72°C for 30 s. The primer sequences were as follows: PPAR*γ* (forward 5′-GGTGAAACTCTGGGAGATTC-3′ and reverse 5′-CAACCATTGGGTCAGCTCTT-3′); C/EBP*α* (forward 5′-AGGTGCTGGAGTTGACCAGT-3′ and reverse 5′-CAGCCTAGAGATCCAGCGAC-3′); GPDH (forward 5′-GAACTAAGGAGCAGCTCAAAGGTTC-3′ and reverse 5′- CAGTTGACTGACTGAGCAAACATAG-3′); *β*-actin (forward 5′-ACCGTGAAAAGATGACCCAG-3′ and reverse 5′-TACGGATGACAACGTCACAC-3′). PCR products were run on 2% agarose gel and then stained with ethidium bromide. Stained bands were visualized under UV light and photographed.

### 2.6. Western Blotting

Whole cell lysates (25 *μ*g) were prepared using lysis buffer (20 mM Tris, pH 7.4, 250 mM NaCl, 2 mM EDTA, pH 8.0, 0.1% Triton X-100, 0.01 mg/mL aprotinin, 0.003 mg/mL leupeptin, 0.4 mM phenylmethylsulfonyl fluoride (PMSF), and 4 mM NaVO4). The lysates were spun at 13000 ×g for 15 min to remove insoluble material and resolved on a 10% SDS-PAGE gel. After electrophoresis, the proteins were electrotransferred to a nitrocellulose membrane, blocked with 5% nonfat milk, and probed with antibodies against PPAR*γ* (Novus, Littleton, CO, USA), C/EBP*α* (Cell Signaling Tech., Danvers, MA, USA), FABP (Cell Signaling Tech., Danvers, MA, USA), and *β*-actin (Sigma, St. Louis, MO, USA) overnight.

The blots were washed, exposed to horseradish peroxidase- (HRP-) conjugated secondary antibodies for 2 h, and finally examined by enhanced chemiluminescence (ECL) (GE Health Care Bio-Sciences, Piscataway, NJ, USA). 

### 2.7. Animals, Diet Manipulation, and EOPK Treatment

Male Sprague-Dawley rats, at 4 weeks of age, were purchased from Hyo-Chang Science (Daegu, Korea) and maintained under conventional conditions. Fifty rats were divided into four groups; normal group (low fat diet), control group (high-fat diet), two EOPK-treated groups- and atorvastatin (positive control) treated group consuming high-fat diets (10 rats per group). Rats were fed the normal (low fat) diet (group 1) or the high-fat diet (groups 2–5) for 6 weeks. High-fat diet composition was described in Table 1. For EOPK treatment, EOPK dissolved in 4% tween 80/normal saline was orally administered once daily to the rats at the doses of 100 (group 3) and 200 mg/kg (group 4) for 6 weeks from the 1st day of high-fat diet feeding, whereas PBS was orally administered to the rats in control group (group 2). As a positive control, atorvastatin was administered at a dose of 10 mg/kg (group 5). 

### 2.8. Preparation of Rat Serum

Whole blood was collected from rats by cardiac puncture method, and serum was isolated by centrifugation at 3000 rpm for 10 min.

### 2.9. Measurement of Total Cholesterol Level

Total cholesterol level was measured by using a total cholesterol assay kit (AM 202-K, Asan Pharm Co., Seoul, Korea) based on Richmond's method [19].

### 2.10. Measurement of Triglyceride Level

Triglyceride level was measured by a triglyceride assay kit (AM 157S-K, Asan Pharm Co., Seoul, Korea) based on McGowan's method [20].

### 2.11. Measurement of Serum HDL and LDL Levels

The levels of high-density lipoprotein (HDL) and low-density lipoprotein (LDL) in serum were measured using Roche cobas C-111 analyzer (Roche-Diagnostics, Indianapolis, IN, USA): AI was calculated by employing the following equation. AI = (total cholesterol − HDL cholesterol)/HDL cholesterol.

### 2.12. Measurement of Body Weight, Retroperitoneal Fat, and Epididymal Fat

The body weight of rats in normal (group 1), control (group 2), EOPK- (100 and 200 mg/kg) treated groups (groups 3 and 4, resp.), and atorvastatin (group 5) was monitored once every week for 6 weeks. The retroperitoneal and epididymal fats were also removed and weighed from rats treated by EOPK (100 and 200 mg/kg) or atorvastatin (10 mg/kg) on the last day of animal study.

### 2.13. Immunohistochemical Staining

For histopathological examination, paraffin sections (4 *μ*m) from tumors dissected were stained with hematoxylin and eosin. Immunohistochemical staining PPAR*γ* (Novus, Littleton, CO, USA) was performed using the indirect avidin/biotin-enhanced horseradish peroxidase method. Antigen retrieval was performed after dewaxing and dehydration of the tissue sections by microwave for 10 min in 10 mM citrate buffer. Sections were cooled to room temperature, treated with 3% hydrogen peroxide in methanol for 10 min, and blocked with 6% horse serum for 30 min at room temperature in humidity chamber. Sections were then incubated with the primary antibody against PPAR*γ* (diluted 1 : 200, Novus, Littleton, CO, USA) at 4°C overnight in humidity chamber. Sections were washed in PBS and incubated with secondary antibody (biotinylated goat anti-rabbit (1 : 150, Vector laboratories, Burlingame, CA, USA) for 30 min in humidity chamber. After further washes, the antibodies were detected with the Vector ABC complex/horseradish peroxidase (HRP) kit (Vector Laboratories, Burlingame, CA, USA) and color-developed with 3,3′-diaminobenzidine tetrahydrochloride. For semiquantitation, ten photomicrographs (200 x) were taken with a CCD camera, avoiding gross necrotic areas. 

### 2.14. Statistical Analyses

All data were expressed as means ± SD. or SE. *In vitro* experiment data were analyzed by Student's *t*-test. *In vivo* experiment data were calculated by the analysis of variance (ANOVA) followed by Duncan's multiple range test. *P* value of less than 0.05 was considered statistically significant. Means in the same column with different superscript letters (a, b, c, d, e, and f) are significantly different (*P* < 0.05) between groups.

## 3. Results

### 3.1. Effect of EOPK on Fat Accumulation in 3T3-L1 Adipocyte-Like Cells

Cytotoxicity of EOPK was determined by MTT assay in 3T3-L1 preadipocytes. Cells were treated with various concentrations of EOPK (0, 12.5, 25, or 50 *μ*g/mL) for 24 h. As shown in Figure 1(a), EOPK had no significant effect on the viability of 3T3-L1 cells. To investigate whether EOPK can affect the cellular differentiation into adipocytes, Oil-Red O staining was performed in 3T3-L1 cells treated with EOPK for 8 days. The differentiated 3T3-L1 adipocytes significantly increased fat accumulation and intracellular triglyceride (Figures 1(b), 1(c), and 1(d)), when compared to preadipocytes. The fat deposits were decreased by 57 and 78% at the treatment with various concentrations of EOPK (25 or 50 *μ*g/mL), respectively, compared to untreated control, adipocytes. Results indicate that 50 *μ*g/mL of EOPK was the most effective ability to inhibit adipocyte differentiation (Figures 1(b) and 1(c)). EOPK treatment reduced the level of triglyceride in cell in a dose-dependent manner (37 and 60% at concentrations of 25 and 50 *μ*g/mL, resp.), compared to preadipocytes (80.04%) (Figure 1(d)).

### 3.2. Effect of EOPK on the Expression of C/EBP, PPAR*γ*, GPDH, and FABP during the Differentiation of Adipocytes

PPAR*γ*, C/EBP*α*, GPDH, and FABP are key factors involved in adipogenesis. In particular, PPAR*γ* controls adipogenic factors as a key transcription factor during adipocyte differentiation. Both mRNA and protein levels of PPAR*γ*, C/EBP*α*, and GPDH were downregulated by EOPK in a dose-dependent manner (Figures 2(a) and 2(b)). To elucidate the underlying mechanism of EOPK, PPAR*γ* antagonist GW9662 was used in 3T3-L1 adipocytes. PPAR*γ* inhibitor GW9662 enhanced the decreased expression of FABP and PPAR*γ* by EOPK (Figure 2(c)).

As shown in Figures 2(d) and 2(e), the lipid accumulation in 3T3-L1 adipocytes treated with EOPK and GW9662 was significantly reduced compared to untreated control. Consistently, immunohistochemistry revealed that EOPK treatment attenuated the expression of PPAR*γ* in the liver tissue sections of EOPK-treated group (100 and 200 mg/kg) compared to untreated control group (Figure 3(c)). Taken together, these results indicate that EOPK inhibits adipocyte differentiation *via* suppressing PPAR**γ**activation.

### 3.3. Effect of EOPK on Body Weight of High-Fat Diet-Fed Rats

The body weights of normal (group 1), control (group 2), EOPK-treated groups (groups 3 and 4), and atorvastatin-treated group (group 5) were monitored once every week for 6 weeks. As shown in Figure 3(a), the body weight of high-fat fed control group was significantly increased 2 weeks after feeding compared to normal low fat group. In contrast, the body weight gain was dose dependently abrogated in EOPK-treated groups, from the date of 3-week treatment of EOPK. Also, six weeks after treatment, the body weight was significantly gained to 331.4 ± 2.8 g in high-fat fed control group compared to normal group (281.6 ± 1.7 g). However, EOPK significantly suppressed the body weights to 309.5 ± 1.8 g and 303.7 ± 2.0 g, respectively, at doses of 100 mg/kg and 200 mg/kg, almost coming up with atorvastatin as positive control (296.5 ± 1.9 g). 

### 3.4. Effects of EOPK on Abdominal Fat Weight of High-Fat Diet-Fed Rats

The retroperitoneal and epididymal fat weight was measured to test whether the body weight normalization by EOPK in high-fat diet-fed rats is associated with a reduction of fat content in body. In the present study, as expected, high-fat diet significantly increased the retroperitoneal fat weight to 18.3 ± 2.91 mg/g from 6.21 ± 1.26 mg/kg body weight. In contrast, EOPK decreased the retroperitoneal fat weight to 15.7 ± 1.86 and 12.7 ± 1.43 mg/g at doses of 100 and 200 mg/kg, respectively, compared to control group (Figure 3(b)). Likewise, epididymal fat weight was also increased in the high-fat diet-fed rats compared to normal group. Oral administration of EOPK decreased epididymal fat pad weight by 10.9 ± 1.85 and 8.52 ± 1.96 mg/g at doses of 100 and 200 mg/kg, respectively (Figure 3(b)).

### 3.5. Effects of EOPK on Serum Lipid and Cholesterol Levels in High-Fat Diet-Fed Rats

The consumption of the high-fat diet significantly increased triglyceride in control group compared to the normal low fat group (Figure 4(a)). EOPK treatment decreased level of serum triglyceride from 131.8 ± 18.2 to 109.3 ± 11.5 and 94.2 ± 8.43 mg/dL at 100 and 200 mg/kg, respectively (Figure 4(a)). Additionally, the consumption of the high-fat diet significantly increased serum total cholesterol compared to the normal low fat group, while EOPK significantly reduced the level of total cholesterol in a dose-dependent manner (Figure 4(b)). The intake of the high-fat diet significantly decreased level of HDL but increased level of LDL compared to normal group (Figure 4(c) control). However, EOPK did not have a significant effect on LDL while elevating HDL level in a dose-dependent manner compared to the high-fat diet control group (Figure 4(c)). Consistently, EOPK treatment significantly decreased the atherosclerosis index (AI) value in a dose-dependent manner compared to the high-fat diet control (Figure 4(d)).

### 3.6. Effects of EOPK on Hepatic Triglyceride and Cholesterol in High-Fat Diet-Fed Rats

The consumption of the high-fat diet significantly increased hepatic triglyceride (Figure 5(a)) and total cholesterol (Figure 5(b)), when compared to the normal low fat group. Oral treatment with EOPK reduced the level of triglyceride from the liver in a dose-dependent manner (24.4 ± 2.47 and 21.2 ± 1.88 mg/g at doses of 100 and 200 mg/kg, resp.), compared to control group (29.8 ± 3.25 mg/g tissue) (Figure 5(a)). In addition, EOPK administration significantly lowered total cholesterol level in liver from 16.9 ± 2.18 mg/g in the high-fat diet control group to 12.6 ± 1.42 and 10.4 ± 1.59 mg/g at 100 and 200 mg/kg, respectively (Figure 5(b)). 

## 4. Discussion

The Korean pine (*P. koraiensis*) is an important afforestation trees in Korea and also distributed in China, Russia, Japan, and Europe [21]. *P. koraiensis *extract attenuated the increase in blood pressure in spontaneously hypertensive rats [13], and its constituent pinolenic acid had cholesterol-lowering effect via regulation of LDL receptor activity in HepG2 hepatoma cells [22]. In addition, *P. koraiensis *nut oil effectively regulated satiety hormones and prospective food intake in postmenopausal overweight women [11]. Our group also reported that essential oil from *P. koraiensis *leaves had antihyperlipidemic effects via upregulation of LDL receptor and inhibition of acyl-coenzyme A: cholesterol acyltransferase [9]. In the current study, we demonstrate that EOPK has antiobesity effects in 3T3-L1 adipocytes and high-fat diet-fed rat models. Adipogenesis is the process of differentiation by which undifferentiated preadipocytes are converted into differentiated adipocytes [23] and subsequently mediate the synthesis and accumulation of lipid [24]. 3T3-L1 cells are the best characterized model to study adipogenesis *in vitro* [25]. Oil-Red O staining revealed that EOPK significantly suppressed fat accumulation and intracellular triglyceride and decreased expression of PPAR*γ*, CEBP*α*, FABP, and GPDH in the differentiated 3T3-L1 adipocytes with no cytotoxicity, indicating the inhibitory effect of EOPK on adipocyte differentiation. Similarly, many natural compounds, including EGCG, berberine, and curcumin, suppressed PPAR*γ* signaling, since PPAR*γ* antagonists have been reported to effectively inhibit adipogenesis and improve insulin sensitivity *in vitro* and *in vivo* [26].

Furthermore, here the antiobesic effect of *P. koraiensis* was confirmed in high-fat diet- (HFD-) treated SD rats at the doses of 100 or 200 mg/kg via blockage of body weight gain. Since loss of body weight is mainly associated with the decrease of fat pad mass as a result of reduction of adipocyte size or triglyceride accumulation [27], our data that EOPK significantly reduced the retroperitoneal and epididymal fat weight and also serum triglyceride compared to HFD fed rats suggest that EOPK can block obesity via inhibition of lipid metabolism including triglyceride. 

Cholesterol is also an important component of fat complex. In particular, low level of serum HDL cholesterol is tightly linked to the occurrence of obesity [28]. In our study, administration of EOPK significantly abrogated the contents of total cholesterol in serum. In addition, EOPK significantly increased level of HDL cholesterol in a dose-dependent manner compared to HFD control group but not LDL cholesterol. Lipid parameters in the blood can be affected by the hepatic metabolisms. As expected, we observed that the hepatic contents of triglyceride and cholesterol were significantly escalated in HFD fed rats compared to normal control. In contrast, EOPK treatment significantly lowered the contents of triglyceride and total cholesterol in the liver, implying that EOPK regulates lipid metabolism including triglyceride and cholesterol against obesity. 

In summary, EOPK inhibited fat accumulation, intracellular triglyceride, and expression of PPAR*γ*, CEBP*α*, FABP, and GPDH in the differentiated 3T3-L1 adipocytes. Also, EOPK attenuated serum and hepatic contents of triglyceride and total cholesterol in HFD fed rat models. Furthermore, EOPK decreased the expression of PPAR*γ* in the liver tissue sections of EOPK-treated rats. Overall, our findings suggest the potential of EOPK as an antiobesity agent.

## Figures and Tables

**Figure 1:** Effect of EOPK on the differentiation of 3T3-L1 adipocytes. (a) Cytotoxicity of EOPK against 3T3-L1 cells was determined by MTT assay. Cells were treated with various concentrations of EOPK (0, 12.5, 25, or 50 *μ*g/mL) for 24 h. (b, c, and d). Confluent cells were treated with 1 *μ*M dexamethasone, 1 *μ*g/mL insulin, and 0.5 mM IBMX for 2 days, and then the medium was replaced by fresh normal medium only containing 1 *μ*g/mL insulin. On day 8, the differentiated adipocyte cells were exposed to EOPK for 2 days. (b) The differentiated cells were stained with Oil-Red O dye and visualized under inverted microscopy at ×100 magnifications. (c) After dissolving and cellular lipid retained Oil-Red O in isopropanol, adipocyte expression was estimated by measuring OD using microplate reader (Sunrise, TECAN, Mannedorf, Switzerland) at 510 nm. (d) Level of intracellular triglyceride.

**Figure 2:** Effects of EOPK on adipocyte differentiation of 3T3-L1 preadipocytes. 3T3-L1 preadipocytes were incubated in medium containing insulin (1.0 *μ*g/mL) with or without the indicated concentrations of EOPK or GW9662. (a) Total RNA was extracted from 3T3-L1 (preadipocytes or adipocytes) cells treated with EOPK and used for RT-PCR analysis of PPAR*γ*, C/EBP*α*, GPDH, and *β*-actin. (b) Total proteins prepared from EOPK-treated 3T3-L1 (preadipocytes or adipocytes) cells were subjected to western blot analysis of PPAR*γ*, C/EBP*α* FABP, and *β*-actin. (c) Total proteins prepared from EOPK- or GW9662-treated 3T3-L1 (preadipocytes or adipocytes) cells were subjected to western blot analysis of PPAR*γ*, FABP, and *β*-actin. (d) Cells were fixed and stained with Oil-Red O. The Oil-Red O-stained adipocytes were photographed at a ×100 magnification under a microscope. (e) Lipids were extracted using isopropanol, and the Oil-Red O was then analyzed at a wavelength of 520 nm. Values are presented as means ± SE. *P < 0.05 versus the control.

**Figure 3:** Effect of EOPK on body and abdominal fat weight of high-fat diet-fed rats. Rats fed a high diet were orally treated with or without EOPK daily for 6 consecutive weeks. (a) Body weights of rats. (b) abdominal fat weights and The retroperitoneal and epididymal fats from rats treated with or without EOPK (100 and 200 mg/kg) were removed and weighed. (c) Representative picture of immunohistochemical staining for PPAR*γ* in liver tissue sections. Data were expressed as means ± SD. Values with the different superscript letters indicate statistical significance (*P* < 0.05) between groups by Duncan's multiple range test.

**Figure 4:** Effects of EOPK on serum lipid and cholesterol levels in high-fat diet-fed rats. (a) Triglyceride level was measured by a triglyceride assay kit (AM 157S-K, Asan Pharm Co., Seoul, Korea). (b) Total cholesterol level was measured by using a total cholesterol assay kit (AM 202-K, Asan Pharm Co., Seoul, Korea). (c) The levels of high-density lipoprotein (HDL) and low-density lipoprotein (LDL) in serum were measured using cobas c 111 analyzer (Roche-Diagnostics, Indianapolis, IN, USA). (d) AI was calculated by employing the following equation: AI = (total cholesterol − HDL cholesterol)/HDL cholesterol. Values with the different superscript letters indicate statistical significance (*P* < 0.05) between groups by Duncan's multiple range test.

**Figure 5:** Effects of EOPK on hepatic triglyceride and cholesterol in high-fat diet-fed rats. The levels of triglyceride (a) and total cholesterol (b) in liver were measured by Biochemistry Analyzer. Values with the different superscript letters indicate statistical significance (*P* < 0.05) between groups by Duncan's multiple range test.

**Table 1:** Composition of basal and high-fat diet.

Ingredient	Basal diet (%)	High-fat diet (%)
Casein	20.0	20.0
DL-Methionine	0.3	0.3
Corn starch	15.0	15.0
Sucrose	50.0	34.5
Fiber^1^	5.0	5.0
Corn oil	5.0	—
AIN-mineral mixture^2^	3.5	3.5
AIN-vitamin mixture^3^	1.0	1.0
Choline bitartrate	0.2	0.2
Beef tallow	—	20.5

^1^Cellulose: Sigma Co. Ltd., USA.

^2^Mineral mixture, based on Rogers and Haper [18], contained the following (g/kg diet): calcium phosphate dibasic 200.0, sodium chloride 74.0, potassium citrate monohydrate 220.0, potassium sulfate 52.0, magnesium oxide 24.0, magnesium carbonate 3.5, ferric citrate 6.0, zinc carbonate 1.6, cupuric carbonate 0.3, potassium iodate 0.01, chromium potassium sulfate 0.55, sucrose, and finely powered make 1,000.

^3^Vitamin mixture (g/kg diet): thiamine HCl 0.6, biotin 0.02, riboflavin 0.6, cyanocobalamin 0.001, pyridoxine HCl 0.7, retinyl acetate 0.8, nicotinic acid 3.0, DL-tocopherol 3.8, Ca-pantothenate 1.6, 7-dehydrocholesterol 0.0025, folic acid 0.2, methionine 0.005, sucrose, and finely powered make 1,000.
